The article "CircTLK1 promotes the proliferation and metastasis of renal cell carcinoma by sponging miR-136-5p" was retracted in 2023. Reason: duplicated images.

# CircTLK1 promotes the proliferation and metastasis of renal cell carcinoma by sponging miR-136-5p

**DOI:** 10.1186/s12943-020-01225-2

**Published:** 2020-06-05

**Authors:** Jianfa Li, Chenchen Huang, Yifan Zou, Jing Ye, Jing Yu, Yaoting Gui

**Affiliations:** 1 Guangdong and Shenzhen Key Laboratory of Male Reproductive Medicine and Genetics, Institute of Urology, Peking University Shenzhen Hospital, Shenzhen-Peking University-the Hong Kong University of Science and Technology Medical Center, Shenzhen, 518000 China; 2 Anhui Medical University, Hefei, 230000 Anhui Province China; 3 Department of Urology, The Affliated Luohu Hospital of Shenzhen University, Shenzhen, 518000 China; 4 Department of Laboratory Medicine, Peking University Shenzhen Hospital, Shenzhen, 518000 China

**Keywords:** Renal cell carcinoma, circTLK1, miR-136-5p, CBX4, VEGFA

## Abstract

**Background:**

Circular RNAs (circRNAs), a novel type of noncoding RNA (ncRNA), are covalently linked circular configurations that form via a loop structure. Accumulating evidence indicates that circRNAs are potential biomarkers and key regulators of tumor development and progression. However, the precise roles of circRNAs in renal cell carcinoma (RCC) remain unknown.

**Methods:**

Through circRNA high-throughput sequencing of RCC cell lines, we identified the circRNA TLK1 (circTLK1) as a novel candidate circRNA derived from the TLK1 gene. qRT-PCR detected the mRNA, circRNA and miRNA expression levels in RCC tissues and cells. Loss-of function experiments were executed to detect the biological roles of circTLK1 in the RCC cell phenotypes in vitro and in vivo. RNA-FISH, RNA pull-down, dual-luciferase reporter, western blot and immunohistochemistry assays were used to investigate the molecular mechanisms underlying the functions of circTLK1.

**Results:**

circTLK1 is overexpressed in RCC, and expression is positively correlated with distant metastasis and unfavorable prognosis. Silencing circTLK1 significantly inhibited RCC cell proliferation, migration and invasion in vitro and in vivo. circTLK1 was mainly distributed in the cytoplasm and positively regulated CBX4 expression by sponging miR-136-5p. Forced CBX4 expression reversed the circTLK1 suppression-induced phenotypic inhibition of RCC cells. Moreover, CBX4 expression was positively correlated with VEGFA expression in RCC tissues. CBX4 knockdown significantly inhibited VEGFA expression in RCC cells.

**Conclusion:**

Collectively, our findings demonstrate that circTLK1 plays a critical role in RCC progression by sponging miR-136-5p to increase CBX4 expression. circTLK1 may act as a diagnostic biomarker and therapeutic target for RCC.

## Introduction

Renal cell carcinoma (RCC) is the second leading cause of death in urologic tumor patients. It is estimated that there were 403,262 new cases of RCC in the world in 2018 [1]. The incidence and mortality of RCC have been rising worldwide﻿ in the past two decades [2]. Approximately 25–30% of RCC patients present with advanced stage disease at first diagnosis, and 30% of localized RCC patients will develop recurrence and metastasis after surgical operation [3]. The 5-year survival rate of advanced stage RCC is extremely low because of resistance to radiation therapy and chemotherapy [4]. Moreover, few RCC biomarkers have been validated. Hence, it is urgent to elucidate the underlying mechanisms in the pathogenesis of RCC and develop effective therapeutic approaches for RCC.

Circular RNAs (circRNAs), a novel type of noncoding RNA (ncRNA), are covalently linked to make up a circular configuration via a connection with the 5′ and 3′ ends [5]. There is growing evidence that circRNAs play important roles in the multilevel regulation of gene expression, including alternative splicing, gene transcription, RNA-protein interactions, and protein-encoding ability [6–8]. However, abnormal expression of circRNAs will cause disorder within the internal environment, thus leading to disease onset or worsening and tumor formation [9, 10]. Emerging studies have suggested that circRNAs are involved in the development of various cancers by regulating various biological processes, including cell growth, differentiation, migration, invasion and apoptosis [11–13]. For instance, circPCNXL2 can promote the proliferation and invasion of RCC cells by regulating the miR-153/ZEB2 axis [14]. circAGFG1 can facilitate the proliferation, migration and invasion of breast cancer cells in vitro and in vivo by regulating the miR-195-5p/CCNE1 axis [15]. circRNA circNOL10 facilitates transcription factor sex comb on midleg-like 1 (SCML1) expression by suppressing transcription factor ubiquitination to inhibit the progression of lung cancer [16]. Several circRNAs were characterized as oncogenes or tumor suppressors in renal RCC [11, 17–19]; however, there are still many circRNAs in RCC, and the roles urgently need to be investigated.

circTLK1 (circbase ID: hsa_circ_0004442), derived from backsplicing the TLK1 mRNA (from exon 9 to exon 10), is located on chromosome 2: 171884848–171,902,872 and is 256 nucleotides (nt) in length. To the best of our knowledge, the function of circTLK1 has not been deeply detected. In this study, we identified that circTLK1 was highly expressed in RCC tissues and positively correlated with distant metastasis and poor prognosis. Silencing of circTLK1 inhibited the proliferation, migration and invasion of RCC cells in vitro and in vivo. Mechanistically, circTLK1 may act as a sponge of miR-136-5p to promote the expression of Chromobox4 (CBX4). Moreover, CBX4 could increase VEGFA expression to facilitate RCC progression. In conclusion, circTLK1 may serve as an oncogene in the progression of RCC and may become an independent prognostic factor for the diagnosis and treatment of RCC.

## Methods

### Patient tissue specimens

A total of 60 RCC tissues and matched adjacent normal tissues were obtained from RCC patients who underwent RCC surgery. This study was approved by the ethical committee of Peking University Shenzhen Hospital. All patients agreed that their samples could be utilized in the experimental studies and publication.

### Cell lines

Human RCC lines (ACHN, 786-O, 769-P, A498, Caki1, and Caki2) were obtained from American Type Culture Collection (ATCC), USA. The human renal epithelial cell lines HK2 and 293 T were purchased from Shanghai Institutes for Biological Sciences, China. The human RCC cell lines were grown in RPMI 1640 medium (Gibco, Carlsbad, CA, USA) supplemented with 10% fetal bovine serum (FBS) (Gibco, South America). The human renal epithelial cell lines were cultured in DMEM (Gibco, Carlsbad, CA, USA) supplemented with 10% FBS. All cells were cultured in a humidified incubator containing 5% CO2 at 37 °C.

### RNA extraction and quantitative real-time PCR

Total RNA from RCC tissues and cell lines was extracted using TRIzol reagent according to the manufacturer’s protocol. The nuclear and cytoplasmic fractions were extracted utilizing NE-PER Nuclear and Cytoplasmic Extraction Reagents (Thermo Scientific, USA). For mRNA and circRNA, total RNAs were reversed by using a reverse transcription kit with a gDNA remover (Toyobo, Japan). For miRNA, cDNA was synthesized by using an All-in-One miRNA Reverse Transcription Kit (GeneCopoeia, Guangzhou, China). Quantification of mRNA and circular RNA was detected by using SYBR Green Real-time PCR Master Mix (Toyobo, Osaka, Japan), and the reactions were performed on a Roche LightCycler® 480II PCR instrument (Basel, Switzerland). GAPDH or U6 was utilized as an internal standard control. The relative RNA expression levels were calculated by the 2^–ΔΔCT^ method. The specific primers used are listed in Additional file 1: Table S1.

### RNase R treatment

RNase R treatment was incubated at 37 °C with 3 U/mg of RNase R (Epicenter, WI, USA) for 30 min in accordance with the manufacturer’s protocol. qRT-PCR was performed to assess the stability of circTLK1 and TLK1 mRNA.

### Cell transfection

Short hairpin RNA (shRNA) targeting circTLK1 or CBX4 was obtained from GenePharma (Suzhou, China). pcDNA3.1-circTLK1, pcDNA-3.1-TLK1 and pcDNA3.1-CBX4 were ordered from GenePharma (Suzhou, China). The miR-136-5p mimic and inhibitor were designed and synthesized by RiboBio (Guangzhou, China). The effects of silencing and overexpression were monitored by RT-PCR. Both oligonucleotides and plasmids were transfected into the RCC cell lines using Lipofectamine 3000 (Invitrogen, USA) according to the manufacturer’s instructions. The sequences of the shRNAs were as follows: shcircTLK1–1: GGACATCTCAAAAAGGCAACA; shcircTLK1–2: CTCAAAAAGGCAACAAGAATG; shTLK1–1: GCAAACCTCCCACAGCTAATA; shTLK1–2: GGATTTCTATCTGAAGCAACA; shCBX4: GATCCGGATGAACCCATAGACTTGTTCAAGAGACAAGTCTATGGGTTCATCCTT TTTTACGCGTG.

### Cell proliferation assay

A CCK-8 assay and a colony-formation assay were used to measure the proliferation of RCC cells. For the CCK-8 assay, the transfected cells were seeded in a 96-well plate for 12 h. The absorbance in each well was measured using a microplate reader (Bio-Rad, USA) at 0, 24, 48 and 72 h. For the colony-formation assay, the transfected RCC cells were cultured in 6-well plates at a density of 1000 cells per well and incubated for 2–3 weeks. Finally, the cells were stained with 0.1% crystal violet and imaged. The stained cells were washed with 33% glacial acetic acid. The absorbance in each well was measured at 550 nm using a microplate reader.

### Cell migration and invasion assays

The migration ability of RCC cells was tested by a wound healing assay and a transwell assay. For the wound healing assay, the transfected cells were seeded in a 6-well plate and grown to 100% confluence. A yellow pipette tip was used to create a clear wound in the cell layer. Images were taken from an optical microscope system at 0 h and 36 h. For the transwell migration assay, the transfected cells were seeded in the upper chambers with 100 μl of serum-free medium, and the lower chamber was filled with medium with 10% FBS. After incubation for 24 h, the cells remaining on the bottom surface of the upper chamber were stained with 0.1% crystal violet solution for 30 min and imaged. The experimental procedure of the transwell invasion assay is similar to that of the transwell migration assay. However, the upper chambers were coated with Matrigel (BD Biosciences, NJ, USA).

### Fluorescence in situ hybridization (FISH)

The fluorescence in situ hybridization assay was conducted to investigate the distribution of circTLK1 in RCC cells by using a Fluorescence in Situ Hybridization Kit (RiboBio, Guangzhou, China). The Cy3-labeled circTLK1 probe was obtained from RiboBio (Guangzhou, China). The Cy3-labeled circTLK1 FISH probe was designated lnc1101096. Images were obtained using a fluorescence microscope.

### Biotin-coupled probe RNA pull-down assay

Biotin-coupled circTLK1 and a negative control probe were designed and synthesized by RiboBio (Guangzhou, China). The sequence of the biotin-coupled circTLK1 probe was CCATTCTTGTTGCCTTTTTG. The sequence of the negative control probe was TTTGCTTGTCTTTTCCCTGA. RCC cells overexpressing circTLK1 were lysed and mixed with a specific circTLK1 probe at 4 °C overnight. The biotin-coupled RNA complex was pulled down by incubating the streptavidin-coated magnetic beads with the cell lysates. The pull-down product was mixed with C-1 magnetic beads (Life Technologies) at 4 °C for 3 h and then washed with wash buffer. The magnetic breads were incubated with proteinase K and lysis buffer to break the formaldehyde cross-links. Finally, the bound RNAs were extracted by using TRIzol for the analysis.

### Luciferase reporter assay

The reporter plasmids (MT06-Firefly_Luciferase-Renilla_Luciferase containing circTLK1 wild-type sequence or mutant sequence and MT06-Firefly_Luciferase-Renilla_Luciferase containing the CBX4 wild-type sequence or mutant sequence) were synthesized by GeneCopoeia (Guangzhou, China). Then, the reporter plasmid and miR-136-5p mimic were cotransfected into RCC cells. The luciferase activities in the transfected cells were measured by using a Dual-Luciferase Reporter Assay System (Promega, WI, USA) after 48 h.

### Western blotting analysis

The protein was extracted from cells using RIPA lysis buffer (Beyotime, China) and quantified using a BCA protein assay kit (Thermo Scientific, USA). Equal amounts of protein were separated by SDS-PAGE gels and transferred onto 0.45 μm PVDF membranes at 330 mA for 70 min. The membranes were blocked by 5% skim milk powder and incubated with a primary antibody at 4 °C overnight, followed by a secondary antibody. Finally, the blots were measured by an enhanced chemiluminescence kit (Millipore, Billerica, USA), and images were obtained by using a BioSpectrum 600 Imaging System (UVP, CA, USA).

### Immunofluorescence and immunohistochemistry

For immunofluorescence, the transfected cells were seeded on glass coverslips for 24 h and then incubated with primary antibodies against E-cadherin/N-cadherin/vimentin (Cell Signaling Technology, USA) at 4 °C overnight. Cell nuclei were counterstained with 2 μg/ml Hoechst for 5 min. Images were captured with a microscope using 20x objectives. For immunohistochemistry, paraffin sections were incubated with primary antibodies against Ki67, CBX4 and VEGFA (Cell Signaling Technology, USA) at 4 °C overnight and then stained with diaminoaniline (DAB).

### Xenografts in mice

The in vivo assay was approved by the animal management committee of Peking University Shenzhen Hospital, and all experimental procedures and animal care were in accordance with the institutional ethics guidelines for animal experiments. For the in vivo tumor formation assay, 10 5-week-old BALB/c nude mice were randomly assigned into the NC group and shRNA-circTLK1 group. Approximately 5× 10^6^ 769-P cells (sh-circTLK1 or shNC) were injected into the backs of nude mice. For rescue experiments in vivo, approximately 1× 10^7^ 769-P cells (sh-circTLK1, shNC or shcircTLK1 + CBX4) were injected into the backs of nude mice. The volume of all xenograft tumors was measured every week by digital calipers. Forty-two days after the injection, the nude mice were sacrificed, and the xenograft tumors were weighed. To create the nude mouse metastasis model, 5-week-old BALB/c nude mice were randomly assigned to the NC group and the shRNA-circTLK1 group. Approximately 2× 10^6^ 769-P cells expressing shcircTLK1 or shNC were injected into the tail veins of nude mice. After 2 months, the nude mice were sacrificed, and the lung metastasis nodules were evaluated by a pathologist. Finally, the lung tissues were removed for hematoxylin-eosin (HE) staining.

### Statistical analysis

The experimental data were analyzed using GraphPad Prism and SPSS 20.0 (IBM, SPSS, Chicago, IL, USA). The differences between groups were analyzed by using Student’s t-test or ANOVA. The Kaplan-Meier method and log-rank test were used to assess the overall survival and disease-free survival curves. Pearson correlation analysis was used to analyze the correlations between groups. A *P* value < 0.05 was considered statistically significant.

## Results

### circTLK1 is overexpressed in RCC tissues and expression is significantly correlated with poor prognosis

To explore the expression profiles of circRNA in RCC, we utilized RNA-seq in normal kidney epithelial cells (293-T) and RCC cells (ACHN, 786-O, 769-P) and discovered that 7335 circRNAs were differentially expressed between normal kidney epithelial cells and RCC cells, among which 1919 circRNAs were upregulated while 5416 circRNAs were downregulated. Ten of the most increased circRNAs are displayed in the heatmap (Fig. 1a). circTLK1 (hsa_circ_0004442) is the most upregulated circRNA among all candidates in 60 pairs of RCC tissue samples (Additional file 2: Fig. S1 a-f). In addition, we investigated the expression of circTLK1 in RCC cells and normal kidney epithelial cells. The data showed that circTLK1 expression in ACHN, 786-O and 769-P cells was significantly higher than the expression in HK2 and 293 T cells (Fig. 1b). CircTLK1 was not only overexpressed in RCC tissues (Fig. 1c) but also highly expressed in RCC patients with postsurgical metastasis (Fig. 1d). In addition, compared to low circTLK1 expression, high circTLK1 expression in RCC patients was negatively associated with a lower overall survival rate (Fig. 1e) and a lower disease-free survival rate (Fig. 1f), suggesting that circTLK1 might be a prognostic tumor marker. circTLK1 was derived from exons 9 and 10 of TLK1 and formed a 247 nt circular transcript according to the CircBase database (http://www.circbase.org/) (Fig. 1g). Further sequence analysis showed that circTLK1 was 247 nt long and contained two exons. Moreover, we found that head-to-tail splicing occurred in the exons from TLK1 by using a divergent primer in cDNA samples and Sanger sequencing (Fig. 1h). The stability of circTLK1 was detected, and the results revealed that RNase R failed to digest circTLK1, but the mRNA expression of TLK1 decreased dramatically after RNase R treatment (Fig. 1i).

**Fig. 1:** circTLK1 is overexpressed in RCC tissues and expression is significantly correlated with poor prognosis. **a** The cluster heat maps show the 10 most increased circRNAs between 293T cells and ACHN, 786-O, and 769-P cells. **b** Relative expression of circTLK1 in RCC cell lines compared to expression in 293T cells. **c** circTLK1 expression in RCC tissues was increased compared to expression in matched normal tissues. **d** circTLK1 expression in RCC patients with no metastasis and distant metastasis. **e** and **f** Kaplan-Meier analysis of the overall survival and disease-free survival of RCC patients with high and low expression of circTLK1. **g** Schematic illustration showing the production of circTLK1 through the circularization of exons 9 and 10 in TLK1. **h** circTLK1 was detected by RT-PCR, and its sequence was proven by Sanger sequencing. The black arrow displays the special splicing junction of circTLK1. **i** Relative expression of circTLK1 and TLK1 in ACHN cells was measured by a qRT-PCR assay upon RNase R treatment. *p < 0.05, **p < 0.01

Compared with HK2, TLK1 expression was significantly downregulated in ACHN, 786-O and 769-P cells (Additional file 3: Fig. S2a). To investigate the function of TLK1 in RCC cells, TLK1 overexpression plasmids or shRNAs targeting TLK1 were transfected into RCC cells. The mRNA and protein expression of TLK1 were significantly increased in RCC cells transfected with pcDNA3.1-TLK1 (Additional file 3: Fig. S2b, c). However, overexpression of TLK1 could not modulate the expression of circTLK1 (Additional file 3: Fig. S2d). The mRNA and protein expression levels of TLK1 were significantly decreased in RCC cells transfected with shTLK1 (Additional file 3: Fig. S2e, f). Suppression of TLK1 did not modulate the expression of circTLK1 (Additional file 3: Fig. S2g). In addition, the results of the CCK-8 and colony-formation assays revealed that forced expression of TLK1 inhibited cell proliferation in the ACHN and 786-O cell lines (Additional file 4: Fig. S3a-d). However, wound healing and transwell invasion assays demonstrated that forced expression of TLK1 could not affect cell mobility and invasion in the ACHN and 786-O cell lines (Additional file 4: Fig. S3e-h).

### circTLK1 knockdown represses RCC cell proliferation

To identify the pathological function of circTLK1 in RCC, we synthesized a shRNA plasmid vector specifically targeting circTLK1 and found that the shRNA vector stably inhibited the expression of circTLK1 in three RCC cell lines (Fig. 2a). Among the shRNAs, shRNA-2 had the best knockdown efficiency. However, suppression of circTLK1 did not change the mRNA (Fig. 2b) and protein (Fig. 2c) expression of TLK1.

**Fig. 2:** circTLK1 knockdown inhibits RCC cell proliferation. **a** qRT-PCR assay was conducted to verify the expression of circTLK1 in RCC cells transfected with two independent shRNAs targeting circTLK1. **b** and **c** The mRNA and protein expression of TLK1 after transfection with shRNA targeting circTLK1. **d** The growth curves of RCC cells transfected with shcircTLK1 were detected by using a CCK-8 assay. **e** and **f** Colony-formation assay was performed to evaluate the proliferation of RCC cells after circTLK1 silencing. *p < 0.05, **p < 0.01, no significant (NS)

We then investigated the effect of circTLK1 on RCC cell proliferation. A CCK-8 assay demonstrated that knockdown of circTLK1 slowed the growth of RCC cells (Fig. 2d). Colony formation assays showed that the colony numbers were obviously reduced after circTLK1 silencing (Fig. 2e, f).

### circTLK1 knockdown inhibits the migration and invasion of RCC cells

Then, wound healing and transwell assays were performed to detect the effects of circTLK1 on the migration and invasion of RCC cells. Our results showed that the migration ability of RCC cells was significantly decreased by circTLK1 downregulation (Fig. 3a-c). In addition, circTLK1 knockdown suppressed RCC cell invasion (Fig. 4d). Based on the role of circTLK1 in the migration and invasion of RCC cells, we suspected that circTLK1 can mediate the epithelial-mesenchymal transition (EMT) process of RCC cells. As shown in Fig. 3e, expression of the mesenchymal markers N-cadherin and vimentin was significantly decreased in circTLK1-silenced cells, while expression of the epithelial marker E-cadherin was increased in circTLK1-suppressed cells. The results of the immunofluorescence assay also confirmed that knockdown of circTLK1 increased expression of E-cadherin and inhibited expression of N-cadherin and vimentin (Additional file 4: Fig. S3 a-c).

**Fig. 3:** circTLK1 knockdown inhibits the migration and invasion of RCC cells. **a** and **b** circTLK1 functions in RCC cell migration as detected with a wound healing assay. **c** circTLK1 functions in RCC cell motility as detected with a transwell assay. **d** circTLK1 functions in RCC cell invasion as detected with a transwell assay. **e** Western blot analysis of the expression of EMT-related proteins (E-cadherin, N-cadherin, and Vimentin) after transfection with shcircTLK1. *p < 0.05, **p < 0.01

**Fig. 4:** circTLK1 acts as a sponge for miR-136-5p in RCC cells. **a** and **b** circTLK1 is mainly located in the cytoplasm of ACHN. **c** circTLK1 in ACHN cells was pulled down by a circTLK1-specific probe and detected by a qRT-PCR assay. **d** miR-136-5p was pulled down by using a circTLK1-specific probe. **e** Schematic illustration of circTLK1-WT and circTLK1-Mut luciferase reporter vectors. **f** Relative luciferase activities were investigated in RCC cells after transfection with circTLK1-WT or circTLK1-Mut and miR-136-5p mimic or miR-NC. **g** and **h** The expression level of miR-136-5p was evaluated by performing a qRT-PCR assay in RCC cells transfected with circTLK1 vector or shcircTLK1. **i** and **j** circTLK1 expression in RCC cells transfected with a miR-136-5p mimic or a miR-136-5p inhibitor. *p < 0.05, **p < 0.01, no significant (NS)

### circTLK1 functions as a miR-136-5p sponge

To elucidate the molecular mechanism underlying circTLK1, we performed FISH and nuclear mass separation assays to detect the subcellular localization of circTL1K. As shown in Fig. 4a, b, we found that circTLK1 was predominantly located in the cytoplasm, indicating that circTLK1 may act as a ceRNA to capture miRNAs, leading to the release of specific miRNA-targeted transcripts. To investigate this hypothesis, we predicted the potential targets of circTLK1 by using the Circular RNA Interactome database (https://circinteractome.nia.nih.gov/). Five potential binding miRNAs were selected, including miR-136-5p, miR-421, miR-659, miR-660-5p and miR-944. Then, an RNA pull-down assay was carried out to evaluate whether circTLK1 could directly capture these candidate miRNAs. The biotinylated circTLK1 probe significantly pulled down circTLK1 in RCC cells upon circTLK1 overexpression (Fig. 4c). Our results showed that miR-136-5p was the only miRNA that was abundantly pulled down by the biotinylated circTLK1 probe in RCC cells (Fig. 4d). In addition, we constructed wild-type (WT) and mutant (Mut) circTLK1 luciferase reporters to detect the role of miR-136-5p in the regulation of circTLK1 activity. After transfection, we observed that overexpression of miR-136-5p significantly inhibited WT circTLK1 luciferase reporter activity but not Mut circTLK1 luciferase reporter activity (Fig. 4e, f). However, overexpression or knockdown of circTLK1 had no effects on the expression of miR-136-5p in RCC cells (Fig. 4g, h). Moreover, overexpression or knockdown of miR-136-5p did not modulate circTLK1 expression in RCC cells (Fig. 4i, j). All these experiments revealed that circTLK1 functioned as a sponge for miR-136-5p.

### miR-136-5p promotes RCC progression by targeting CBX4

Based on the interaction between circTLK1 and miR-136-5p, we explored the potential roles of miR-136-5p in RCC. A previous study indicated that miR-136-5p acted as a tumor suppressor in the progression of RCC, inhibiting the proliferation, migration and invasion of RCC cells [20]. Furthermore, miRNAs can regulate the expression of their target mRNA by binding to the 3’UTR of the mRNA. To identify the potential genes of miR-136-5p, we conducted bioinformatics analysis by using the TargetScan, miRDB, Starbase and miRTarBase databases and selected CBX4, GNAS, LUZP6, MSL2, MTMR4 and SOCS7 as the potential targets of miR-136-5p (Fig. 5a). Further comprehensive transcriptional analysis with our dataset demonstrated that miR-136-5p expression was negatively correlated with CBX4 expression (Fig. 5b). To investigate whether CBX4 was a possible target of miR-136-5p, a WT or Mut sequence of the 3’UTR of CBX4 containing the miR-136-5p-binding sequence was employed to synthesize a luciferase reporter plasmid (Fig. 5c). The results of luciferase reporter analysis showed that cotransfection of a miR-136-5p mimic and a CBX4 WT plasmid strongly decreased the luciferase activity. However, cotransfection of a miR-136-5p mimic and a CBX4 Mut plasmid did not change the luciferase activity (Fig. 5d). Moreover, forced expression of miR-136-5p inhibited the mRNA and protein expression of CBX4 (Fig. 5e-g). Next, we detected the role of CBX4 in the progression of RCC. As shown in Fig. 5h, CBX4 expression in RCC tissues was upregulated compared to that in normal tissues. We found that CBX4 expression was positively correlated with tumor size and postoperative metastasis (Fig. 5i, j). In addition, high expression of CBX4 in RCC patients was associated with a lower overall survival rate than low expression of CBX4 (Fig. 5k).

**Fig. 5:** CBX4 is a direct target of miR-136-5p. **a** Schematic illustration exhibiting the overlap between the target mRNAs and miR-136-5p as predicted by TargetScan, miRDB, Starbase and miRTarBase. **b** Comprehensive transcriptional analysis indicated that miR-136-5p expression was negatively correlated with CBX4 expression in RCC tissues. **c** Schematic illustration of CBX4-WT and CBX4 Mut luciferase reporter vectors. **d** Relative luciferase activities were measured in RCC cells after transfection with CBX4-WT or CBX4 Mut and a miR-136-5p mimic or miR-NC. **e** CBX4 mRNA expression was evaluated by performing qRT-PCR assays in RCC cells transfected with a miR-136-5p mimic. **f** and **g** CBX4 protein expression was detected by performing western blot and immunofluorescence assays in RCC cells transfected with a miR-136-5p mimic. **h** CBX4 expression was increased in RCC tissues compared to matched normal tissues. **i** CBX4 expression in RCC patients with different tumor sizes. **j** CBX4 expression in RCC patients with no metastasis or distant metastasis. **k** Kaplan-Meier analysis of the overall survival of RCC patients with high and low expression of CBX4. *p < 0.05, **p < 0.01, no significant (NS)

### CBX4 knockdown inhibits the proliferation, migration and invasion of RCC cells

We next investigated the roles of CBX4 in RCC cell phenotypes. Using shRNA targeting circTLK1, we effectively repressed its expression in ACHN and 769-P cells (Fig. 6a). Through a CCK-8 assay, we discovered that silencing CBX4 significantly suppressed the proliferation of ACHN and 769-P cells (Fig. 6b, c). The colony-formation assay also illustrated that knockdown of CBX4 greatly impaired the proliferation ability of RCC cells (Fig. 6d, e). Further experiments showed that silencing CBX4 significantly inhibited the migration and invasion of ACHN and 769-P cells (Fig. 6f-i). Moreover, we identified that the CBX4 mRNA level was positively correlated with the VEGFA mRNA level in The Cancer Genome Atlas (TCGA) database and our dataset (Fig. 6j). CBX4 knockdown inhibited the mRNA and protein levels of VEGFA (Fig. 6k).

**Fig. 6:** CBX4 knockdown inhibits the proliferation, migration and invasion of RCC cells. **a** qRT-PCR assay was conducted to verify the expression of CBX4 in RCC cells transfected with shRNA targeting CBX4. **b** and **c** The growth curves of RCC cells transfected with shCBX4 were detected by using a CCK-8 assay. **d** and **e** Colony-formation assays were performed to measure the proliferation of RCC cells after CBX4 silencing. **f** and **g** Cell migration was examined in RCC cells transfected with shCBX4 or shNC by a wound healing assay. **h** and **i** Cell invasion was detected in RCC cells transfected with shCBX4 or shNC by a transwell assay. **j** Comprehensive transcriptional analysis indicated that CBX4 expression was significantly positively correlated with VEGFA expression in RCC tissues. **k** Knockdown of CBX4 suppressed the mRNA and protein expression of VEGFA. *p < 0.05, **p < 0.01

### CBX4 overexpression reverses the inhibitory effect of circTLK1 suppression on cell proliferation and metastasis

To explore whether circTLK1 exerts its biological function by regulating CBX4 expression, a rescue assay between circTLK1 and CBX4 was performed. We found that knockdown of circTLK1 obviously inhibited the mRNA and protein expression of CBX4 (Fig. 7a, b). A CCK-8 assay revealed that CBX4 overexpression significantly reversed the circTLK1 suppression-induced growth curve inhibition in ACHN and 769-P cells (Fig. 7c). Colony formation assays showed that forced expression of CBX4 reversed the circTLK1 silencing-induced cell proliferation inhibition (Fig. 7d, e). In addition, CBX4 upregulation significantly reversed the cell migration (Fig. 7f-i) and invasion (Fig. 7j, k) suppression of RCC cells induced by circTLK1 silencing.

**Fig. 7:** CBX4 overexpression reverses the shcircTLK1-induced decrease in cell proliferation, migration and invasion in RCC cells. **a** and **b** Knockdown of circTLK1 inhibited the mRNA and protein expression of CBX4. **c**-**e** Overexpression of CBX4 reversed circTLK1 silencing-induced cell proliferation inhibition. **f**-**i** Overexpressing CBX4 significantly reversed circTLK1 silencing-induced cell migration suppression. **j** and **k** Augmented expression of CBX4 significantly reversed circTLK1 silencing-induced cell invasion inhibition. *p < 0.05, **p < 0.01

### circTLK1 knockdown inhibits the growth and metastasis of RCC cells in vivo

To investigate the role of circTLK1 in the growth and lung metastasis of RCC in vivo, stable 769-P cells transfected with shcircTLK1 or shNC were injected into nude mice to establish a xenograft tumor and a lung metastasis nude mouse model. In the xenograft tumor model, the tumors derived from cells transfected with shcircTLK1 were smaller than those derived from cells transfected with shNC (Fig. 8a). Knockdown of circTLK1 significantly suppressed the tumor volume and weight (Fig. 8b-c). Furthermore, knockdown of circTLK1 inhibited the mRNA expression of CBX4 and VEGFA in vivo (Fig. 8d). IHC assays suggested that decreased expression of circTLK1 inhibited the expression of Ki67, CBX4 and VEGFA (Fig. 8e). In the lung metastasis nude mouse model, suppression of circTLK1 led to a notable decrease in metastasis in the lungs (Fig. 8f-g). Further, HE staining revealed fewer lung tumor foci in the shcircTLK1 group than in the shNC group (Fig. 8h). Moreover, the xenograft tumor model showed that overexpression of CBX4 reversed circTLK1 silencing-induced cell growth inhibition (Fig. 8i-k). This in vivo study demonstrated that circTLK1 may play an important role in promoting the growth and metastasis of RCC in vivo. In general, we illustrated that circTLK1 contributed to RCC growth and metastasis by sponging miR-513a-5p to modulate CBX4 expression (Fig. 8l).

**Fig. 8:** circTLK1 knockdown inhibits tumorigenesis and lung metastasis of RCC cells in vivo. **a** Xenograft tumor models showed that tumors grown from the shcircTLK1 group were smaller than those grown from the shNC group (*n*=5). **b** and **c** Compared with the shNC group, the shcircTLK1 group had tumors with significantly decreased volume and weight. **d** Knockdown of circTLK1 inhibited the mRNA expression of CBX4 and VEGFA in vivo. **e** An IHC assay was performed to evaluate the protein expression of Ki67, CBX4 and VEGFA. **f** Representative images of the mouse lungs after transplantation for 8 weeks. **g** The number of lung metastases in each group. **h** HE staining of metastatic nodules of the lungs. **i**-**k** Xenograft tumor model showed that forced expression of CBX4 reversed the cell growth inhibition induced by silencing circTLK1. **l** Schematic diagram displaying the mechanism underlying circTLK1 as a ceRNA for miR-136-5p. *p < 0.05, **p < 0.01

## Discussion

High-throughput sequencing has demonstrated that only 2% of the whole human genome can be translated into proteins, while the remaining 98% can be transcribed into only noncoding RNAs that do not have coding potential [21]. Noncoding RNAs are classified as miRNAs, small nuclear RNAs (snRNAs), lncRNAs (long noncoding RNAs) and circRNAs. There is no doubt that lncRNAs and circRNAs have attracted increasing attention in cancer research [22–24]. LncRNAs are generally described as RNA transcripts of more than 200 nt in length without protein-coding potential. LncRNAs are transcribed by RNA polymerase II, owing to a 5′-cap and 3′-polyA tail [25]. LncRNAs localized in the nucleus are involved in chromatin interactions, RNA processing and transcriptional regulation, while cytoplasmic lncRNAs serve as “miRNA sponges” to reverse the negative effects of miRNAs on their target genes. Moreover, lncRNAs exert their biological functions during cellular processes, including acting as transcriptional regulators, miRNA sponges, molecular bait and protein complex scaffolds [26, 27]. Another novel type of noncoding RNA is circRNA, which is created by a noncanonical splicing process named backsplicing and is transcribed by RNA polymerase II. Unlike linear RNAs, circRNAs are covalently linked to make closed circular transcripts via a connection between the 5′ and 3′ ends [28]. Hence, circRNAs lack a 5′-cap and 3′-polyA tail, which makes them resistant to RNase R treatment. CircRNAs exert their biological functions during cellular processes, including acting as miRNA and protein sponges and modulating parental gene transcription and protein translation [29, 30].

In recent years, with the development of RNA sequencing (RNA-seq) and circRNA-specific bioinformatics technology, circRNAs have been found to be expressed at low levels and display cell-type specific, tissue-specific and organism-specific patterns. Accumulating evidence has revealed that circRNAs are involved in the occurrence and progression of various diseases, including neurological disorders, cardiovascular system diseases, osteoarthritis and cancers [31–34]. In particular, circRNAs play important roles in tumor initiation, growth and metastasis. A previous study suggested that circRNAs could regulate the malignant phenotype of RCC by serving as endogenous competitive RNAs in the development of RCC. For example, circAKT3 suppresses the metastasis of clear cell RCC by modulating miR-296-3p/E-cadherin signals. Further, circPCNXL2 can facilitate the proliferation and invasion of RCC cells by modulating the miR-153/ZEB2 axis. Finally, circRNAZNF609 sponges miR-138-5p to promote the proliferation and invasion of RCC cells by increasing FOXP4 expression. However, the function and mechanism of circRNAs in RCC are still mysterious.

In this study, we performed RNA-seq to obtain the expression profiles of circRNAs in RCC cells and 293 T cells. Subsequently, we identified a novel circRNA termed circTLK1 that was significantly upregulated in RCC tissues and positively correlated with distant metastasis and poor prognosis. circTLK1 is derived from exons 9 and 10 of its host gene TLK1, which is a known kinase in prostate cancer and may regulate DNA repair, replication and chromosome segregation [35, 36]. Silencing of circTLK1 had no effects on the mRNA and protein expression of TLK1, indicating that circTLK1 does not encode a protein. In addition, overexpression or knockdown of TLK1 could not modulate the expression of TLK1. Further experiments showed that knockdown of circTLK1 suppressed the proliferation and metastatic abilities of RCC cells in vitro and in vivo. These results suggest that circTLK1 plays an important role in the pathogenesis and development of RCC.

The ceRNA hypothesis states that RNA transcripts, including lncRNAs, circRNAs, pseudogene transcripts and mRNAs, could regulate the expression of target genes by interacting with miRNAs [37–39]. They usually competitively bind to miRNA response elements (MREs) to regulate mRNA expression, building a complex posttranscriptional regulatory network [40]. A growing body of evidence suggests that some circRNAs can act as miRNA sponges to modulate miRNA target gene expression in various cancers. For example, it was reported that circPRMT5 promoted the EMT process in bladder cancer by acting as a sponge for miR-30c to regulate the expression of E-cadherin and snail [41]. In addition, circMTO1 inhibits the proliferation of hepatocellular carcinoma by sponging miR-9 as a ceRNA and reverses its inhibition of p21, its target gene [42]. Moreover, circSLC8A1 functions as a sponge for miR-130b and miR-494 to suppress proliferation, migration and invasion of bladder cancer cells [43]. In our study, FISH and nuclear mass separation assays showed that circTLK1 was mainly located in the cytoplasm of RCC cells. RNA pull-down and dual-luciferase reporter assays confirmed that circTLK1 could directly bind to miR-136-5p. In addition, overexpression or knockdown of circTLK1 could not modulate miR-136-5p expression in RCC cells, suggesting that circTLK1 functions as a “miRNA sponge” of miR-136-5p. As a competing endogenous RNA, circTLK1 could not affect the total expression of miR-136-5p but could affect only the unbound form of miR-136-5p. That is, circTLK1 fails to degrade miR-136-5p at the posttranscriptional level. CDR1a, a well-known circRNA, contains 63 conserved binding sites for miR-7. CDR1a can directly sponge miR-7 with its MREs and suppress the activity of miR-7. However, CDR1a could not regulate the total expression of miR-7 [44]. It has been reported that miR-136-5p is significantly downregulated in RCC tissues. Forced expression of miR-136-5p significantly inhibited cell proliferation, migration and invasion and induced apoptosis of RCC cells [20]. miR-136-5p is also expressed at low levels and acts as a tumor suppressor in the progression of other cancers, including gallbladder and ovarian cancer [45, 46]. Our data suggested that circTLK1 acted as an oncogene by acting as a sponge in RCC and revealed the relationship between circTLK1 and miR-136-5p during the tumorigenesis and progression of RCC.

Based on the ceRNA hypothesis, circRNA could serve as a ceRNA to regulate the expression of miRNA target genes. Bioinformatics analysis revealed that CBX4 was a potential target of miR-136-5p. Further dual-luciferase reporter assays demonstrated that miR-136-5p directly bound to the 3’UTR of CBX4. Moreover, overexpression of miR-136-5p obviously inhibited the mRNA and protein expression of CBX4. CBX4 (also called polycomb 2, Pc2), a small ubiquitin-related modifier (SUMO) E3 ligase, can facilitate the sumoylation of other proteins involved in ﻿tumorigenesis, such as the DNA methyltransferase Dnmt3a and BMI1 [47, 48]. In hepatocellular carcinoma, upregulation of CBX4 is positively correlated with histological grade, tumor-node-metastasis stage and distant metastasis [49]. Mechanistically, CBX4 can increase VEGFA expression and angiogenesis in HCC cells by promoting the sumoylation of HIF-1a [50]. In breast cancer, CBX4 promotes cell growth and metastasis in vitro and in vivo by regulating the miR-137/Notch1 signaling pathway [51]. In our study, we found that CBX4 was upregulated in RCC tissues and positively correlated with tumor size, distant metastasis and poor prognosis. Knockdown of CBX4 suppressed the proliferation, migration and invasion of RCC cells. Consistent with the results of previous studies, decreased CBX4 expression inhibited VEGFA mRNA and protein expression. To validate the crosstalk between circTLK1 and CBX4, we discovered that attenuated circTLK1 expression could decrease CBX4 at both the mRNA and protein levels. Furthermore, upregulation of CBX4 abolished the inhibitory effect of circTLK1 suppression on cell proliferation and metastasis, which might support our hypothesis that circTLK1 acts as a ceRNA to facilitate CBX4-mediated proliferation and metastasis by absorbing miR-136-5p in RCC.

## Conclusions

In conclusion, we identified the novel circRNA circTLK1 that plays an oncogenic role in RCC and is correlated with poor prognosis. Further experiments demonstrated that circTLK1 might sponge miR-136-5p to regulate circTLK1 expression, promoting the tumorigenesis and development of RCC. Our results revealed that circTLK1 might serve as a future prognostic marker and therapeutic target for RCC. The regulatory network involving the circTLK1/miR-136-5p/CBX4/VEGFA axis might provide new insight into the potential mechanism of the pathogenesis and development of RCC.

## Supplementary information

**Additional file 1: Table S1.** The primer sequences included in this study.

**Additional file 2: Figure S1.** Relative expression of six alternative circular RNAs in 60 pairs of RCC tissue samples. a-f Relative expression of circRNA_0003731, circRNA_0004442, circRNA_0004087, circRNA_0005239, circRNA_0003271 and circRNA_0005081 in 60 RCC tissues and matched adjacent normal tissues by a qRT-PCR assay. *p < 0.05, **p < 0.01.

**Additional file 3: Figure S2.** The correlation between TLK1 expression and circTLK1 expression in RCC cells. a TLK1 in RCC cells was upregulated compared with that in HK2 cells. b and c The mRNA and protein expression of TLK1 were increased significantly in RCC cells transfected with a pcDNA-3.1 TLK1 vector. d Overexpression of TLK1 could not modulate circTLK1 expression in RCC cells. e and f The mRNA and protein expression of TLK1 were obviously decreased in RCC cells transfected with shRNAs targeting TLK1. g Knockdown of TLK1 could not modulate circTLK1 expression in RCC cells. *p < 0.05, **p < 0.01, no significant (NS).

**Additional file 4: Figure S3.** TLK1 overexpression inhibits the proliferation of RCC cells. a and b The growth curves of RCC cells transfected with pcDNA3.1-TLK1 were measured by a CCK-8 assay. c and d The colony-formation abilities of RCC cells transfected with pcDNA3.1-TLK1 were measured by a colony-formation assay. e and f Overexpression of TLK1 did not change the migration capacity of RCC cells transfected with pcDNA3.1-TLK1. g and h Overexpression of TLK1 did not change the invasion capacity of RCC cells transfected with pcDNA3.1-TLK1. *p < 0.05, **p < 0.01, no significant (NS).

**Additional file 5: Figure S4.** circTLK1 knockdown inhibits the EMT process of RCC cells. a-c Suppression of circTLK1 increased the expression of E-cadherin and inhibited the expression of N-cadherin and vimentin in RCC cells.

## Data Availability

The datasets supporting the conclusions of this article are included within the article and its Additional files.

## Abbreviations

RCC: Renal cell carcinoma
circRNA: Circular RNA
circTLK1: Circular RNA TLK1
RNA-seq: RNA sequencing
qRT-PCR: Quantitative real-time PCR
shRNA: Short hairpin RNA
ceRNA: Competing endogenous RNA
FBS: Fetal bovine serum
FISH: Fluorescence in situ hybridization
HE: Hematoxylin-eosin
EMT: Epithelial-mesenchymal transition
MREs: MiRNA response elements
WT: Wild type
Mut: Mutant
NS: No significant

## References

[1] Bray F, Ferlay J, Soerjomataram I, Siegel RL, Torre LA, Jemal A (2018). Global cancer statistics 2018: GLOBOCAN estimates of incidence and mortality worldwide for 36 cancers in 185 countries. CA Cancer J Clin.

[2] Capitanio U, Montorsi F (2016). Renal cancer. Lancet.

[3] Choueiri TK, Motzer RJ (2017). Systemic therapy for metastatic renal-cell carcinoma. N Engl J Med.

[4] Topalian SL, Hodi FS, Brahmer JR, Gettinger SN, Smith DC, McDermott DF, Powderly JD, Sosman JA, Atkins MB, Leming PD, Spigel DR, Antonia SJ, Drilon A, Wolchok JD, Carvajal RD, McHenry MB, Hosein F, Harbison CT, Grosso JF, Sznol M (2019). Five-year survival and correlates among patients with advanced melanoma, renal cell carcinoma, or non-small cell lung cancer treated with Nivolumab. JAMA Oncol.

[5] Hentze MW, Preiss T (2013). Circular RNAs: splicing’s enigma variations. EMBO J.

[6] Dong Y, He D, Peng Z, Peng W, Shi W, Wang J, Li B, Zhang C, Duan C (2017). Circular RNAs in cancer: an emerging key player. J Hematol Oncol.

[7] Zhang Y, Xue W, Li X, Zhang J, Chen S, Zhang JL, Yang L, Chen LL (2016). The biogenesis of nascent circular RNAs. Cell Rep.

[8] Chen LL (2016). The biogenesis and emerging roles of circular RNAs. Nat Rev Mol Cell Biol.

[9] Chen Y, Li C, Tan C, Liu X (2016). Circular RNAs: a new frontier in the study of human diseases. J Med Genet.

[10] Boon RA, Jae N, Holdt L, Dimmeler S (2016). Long noncoding RNAs: from clinical genetics to therapeutic targets?. J Am Coll Cardiol.

[11] Xue D, Wang H, Chen Y, Shen D, Lu J, Wang M, Zebibula A, Xu L, Wu H, Li G, Xia L (2019). Circ-AKT3 inhibits clear cell renal cell carcinoma metastasis via altering miR-296-3p/E-cadherin signals. Mol Cancer.

[12] Li X, Ding J, Wang X, Cheng Z, Zhu Q. NUDT21 regulates circRNA cyclization and ceRNA crosstalk in hepatocellular carcinoma. Oncogene. 2019;39:891–904.10.1038/s41388-019-1030-031570791

[13] Huang C, Deng H, Wang Y, Jiang H, Xu R, Zhu X, Huang Z, Zhao X (2019). Circular RNA circABCC4 as the ceRNA of miR-1182 facilitates prostate cancer progression by promoting FOXP4 expression. J Cell Mol Med.

[14] Zhou B, Zheng P, Li Z, Li H, Wang X, Shi Z, Han Q (2018). CircPCNXL2 sponges miR-153 to promote the proliferation and invasion of renal cancer cells through upregulating ZEB2. Cell Cycle.

[15] Yang R, Xing L, Zheng X, Sun Y, Wang X, Chen J (2019). The circRNA circAGFG1 acts as a sponge of miR-195-5p to promote triple-negative breast cancer progression through regulating CCNE1 expression. Mol Cancer.

[16] Nan A, Chen L, Zhang N, Jia Y, Li X, Zhou H, Ling Y, Wang Z, Yang C, Liu S, Jiang Y (2019). Circular RNA circNOL10 inhibits lung cancer development by promoting SCLM1-mediated transcriptional regulation of the Humanin polypeptide family. Adv Sci (Weinh).

[17] Chen Q, Liu T, Bao Y, Zhao T, Wang J, Wang H, Wang A, Gan X, Wu Z, Wang L (2019). CircRNA cRAPGEF5 inhibits the growth and metastasis of renal cell carcinoma via the miR-27a-3p/TXNIP pathway. Cancer Lett.

[18] Han Z, Zhang Y, Sun Y, Chen J, Chang C, Wang X, Yeh S (2018). ERbeta-mediated alteration of circATP2B1 and miR-204-3p signaling promotes invasion of clear cell renal cell carcinoma. Cancer Res.

[19] Wang K, Sun Y, Tao W, Fei X, Chang C (2017). Androgen receptor (AR) promotes clear cell renal cell carcinoma (ccRCC) migration and invasion via altering the circHIAT1/miR-195-5p/29a-3p/29c-3p/CDC42 signals. Cancer Lett.

[20] Chen P, Zhao L, Pan X, Jin L, Lin C, Xu W, Xu J, Guan X, Wu X, Wang Y, Yang S, Wang T, Lai Y (2018). Tumor suppressor microRNA-136-5p regulates the cellular function of renal cell carcinoma. Oncol Lett.

[21] Birney E, Stamatoyannopoulos JA, Dutta A, Guigo R, Gingeras TR, Margulies EH, Weng Z, Snyder M, Dermitzakis ET, Thurman RE, Kuehn MS, Taylor CM, Neph S, Koch CM, Asthana S, Malhotra A, Adzhubei I, Greenbaum JA, Andrews RM, Flicek P, Boyle PJ, Cao H, Carter NP, Clelland GK, Davis S, Day N, Dhami P, Dillon SC, Dorschner MO, Fiegler H, Giresi PG, Goldy J, Hawrylycz M, Haydock A, Humbert R, James KD, Johnson BE, Johnson EM, Frum TT, Rosenzweig ER, Karnani N, Lee K, Lefebvre GC, Navas PA, Neri F, Parker SC, Sabo PJ, Sandstrom R, Shafer A, Vetrie D, Weaver M, Wilcox S, Yu M, Collins FS, Dekker J, Lieb JD, Tullius TD, Crawford GE, Sunyaev S, Noble WS, Dunham I, Denoeud F, Reymond A, Kapranov P, Rozowsky J, Zheng D, Castelo R, Frankish A, Harrow J, Ghosh S, Sandelin A, Hofacker IL, Baertsch R, Keefe D, Dike S, Cheng J, Hirsch HA, Sekinger EA, Lagarde J, Abril JF, Shahab A, Flamm C, Fried C, Hackermuller J, Hertel J, Lindemeyer M, Missal K, Tanzer A, Washietl S, Korbel J, Emanuelsson O, Pedersen JS, Holroyd N, Taylor R, Swarbreck D, Matthews N, Dickson MC, Thomas DJ, Weirauch MT, Gilbert J, Drenkow J, Bell I, Zhao X, Srinivasan KG, Sung WK, Ooi HS, Chiu KP, Foissac S, Alioto T, Brent M, Pachter L, Tress ML, Valencia A, Choo SW, Choo CY, Ucla C, Manzano C, Wyss C, Cheung E, Clark TG, Brown JB, Ganesh M, Patel S, Tammana H, Chrast J, Henrichsen CN, Kai C, Kawai J, Nagalakshmi U, Wu J, Lian Z, Lian J, Newburger P, Zhang X, Bickel P, Mattick JS, Carninci P, Hayashizaki Y, Weissman S, Hubbard T, Myers RM, Rogers J, Stadler PF, Lowe TM, Wei CL, Ruan Y, Struhl K, Gerstein M, Antonarakis SE, Fu Y, Green ED, Karaoz U, Siepel A, Taylor J, Liefer LA, Wetterstrand KA, Good PJ, Feingold EA, Guyer MS, Cooper GM, Asimenos G, Dewey CN, Hou M, Nikolaev S, Montoya-Burgos JI, Loytynoja A, Whelan S, Pardi F, Massingham T, Huang H, Zhang NR, Holmes I, Mullikin JC, Ureta-Vidal A, Paten B, Seringhaus M, Church D, Rosenbloom K, Kent WJ, Stone EA, Batzoglou S, Goldman N, Hardison RC, Haussler D, Miller W, Sidow A, Trinklein ND, Zhang ZD, Barrera L, Stuart R, King DC, Ameur A, Enroth S, Bieda MC, Kim J, Bhinge AA, Jiang N, Liu J, Yao F, Vega VB, Lee CW, Ng P, Shahab A, Yang A, Moqtaderi Z, Zhu Z, Xu X, Squazzo S, Oberley MJ, Inman D, Singer MA, Richmond TA, Munn KJ, Rada-Iglesias A, Wallerman O, Komorowski J, Fowler JC, Couttet P, Bruce AW, Dovey OM, Ellis PD, Langford CF, Nix DA, Euskirchen G, Hartman S, Urban AE, Kraus P, Van Calcar S, Heintzman N, Kim TH, Wang K, Qu C, Hon G, Luna R, Glass CK, Rosenfeld MG, Aldred SF, Cooper SJ, Halees A, Lin JM, Shulha HP, Zhang X, Xu M, Haidar JN, Yu Y, Ruan Y, Iyer VR, Green RD, Wadelius C, Farnham PJ, Ren B, Harte RA, Hinrichs AS, Trumbower H, Clawson H, Hillman-Jackson J, Zweig AS, Smith K, Thakkapallayil A, Barber G, Kuhn RM, Karolchik D, Armengol L, Bird CP, de Bakker PI, Kern AD, Lopez-Bigas N, Martin JD, Stranger BE, Woodroffe A, Davydov E, Dimas A, Eyras E, Hallgrimsdottir IB, Huppert J, Zody MC, Abecasis GR, Estivill X, Bouffard GG, Guan X, Hansen NF, Idol JR, Maduro VV, Maskeri B, McDowell JC, Park M, Thomas PJ, Young AC, Blakesley RW, Muzny DM, Sodergren E, Wheeler DA, Worley KC, Jiang H, Weinstock GM, Gibbs RA, Graves T, Fulton R, Mardis ER, Wilson RK, Clamp M, Cuff J, Gnerre S, Jaffe DB, Chang JL, Lindblad-Toh K, Lander ES, Koriabine M, Nefedov M, Osoegawa K, Yoshinaga Y, Zhu B, de Jong PJ, E.P. Consortium, N.C.S. Program, C. Baylor College of Medicine Human Genome Sequencing, C. Washington University Genome Sequencing, I. Broad, I. Children’s Hospital Oakland Research (2007). Identification and analysis of functional elements in 1% of the human genome by the ENCODE pilot project. Nature.

[22] Wang X, Yang J, Guo G, Feng R, Chen K, Liao Y, Zhang L, Sun L, Huang S, Chen JL (2019). Novel lncRNA-IUR suppresses Bcr-Abl-induced tumorigenesis through regulation of STAT5-CD71 pathway. Mol Cancer.

[23] Kong Y, Li Y, Luo Y, Zhu J, Zheng H, Gao B, Guo X, Li Z, Chen R, Chen C (2020). circNFIB1 inhibits lymphangiogenesis and lymphatic metastasis via the miR-486-5p/PIK3R1/VEGF-C axis in pancreatic cancer. Mol Cancer.

[24] Li J, Huang C, Zou Y, Yu J, Gui Y. Circular RNA MYLK promotes tumour growth and metastasis via modulating miR-513a-5p/VEGFC signalling in renal cell carcinoma. J Cell Mol Med. 2020;00:1–13.10.1111/jcmm.15308PMC729968932342645

[25] Yao RW, Wang Y, Chen LL (2019). Cellular functions of long noncoding RNAs. Nat Cell Biol.

[26] Huarte M (2015). The emerging role of lncRNAs in cancer. Nat Med.

[27] Schmitt AM, Chang HY (2016). Long noncoding RNAs in cancer pathways. Cancer Cell.

[28] Kristensen LS, Andersen MS, Stagsted LVW, Ebbesen KK, Hansen TB, Kjems J (2019). The biogenesis, biology and characterization of circular RNAs. Nat Rev Genet.

[29] Sun J, Li B, Shu C, Ma Q, Wang J (2020). Functions and clinical significance of circular RNAs in glioma. Mol Cancer.

[30] Shang Q, Yang Z, Jia R, Ge S (2019). The novel roles of circRNAs in human cancer. Mol Cancer.

[31] Bai Y, Zhang Y, Han B, Yang L, Chen X, Huang R, Wu F, Chao J, Liu P, Hu G, Zhang JH, Yao H (2018). Circular RNA DLGAP4 ameliorates ischemic stroke outcomes by targeting miR-143 to regulate endothelial-mesenchymal transition associated with blood-brain barrier integrity. J Neurosci.

[32] Garikipati VNS, Verma SK, Cheng Z, Liang D, Truongcao MM, Cimini M, Yue Y, Huang G, Wang C, Benedict C, Tang Y, Mallaredy V, Ibetti J, Grisanti L, Schumacher SM, Gao E, Rajan S, Wilusz JE, Goukassian D, Houser SR, Koch WJ, Kishore R (2019). Circular RNA CircFndc3b modulates cardiac repair after myocardial infarction via FUS/VEGF-A axis. Nat Commun.

[33] Zhou ZB, Huang GX, Fu Q, Han B, Lu JJ, Chen AM, Zhu L (2019). circRNA.33186 contributes to the pathogenesis of osteoarthritis by sponging miR-127-5p. Mol Ther.

[34] Kristensen LS, Hansen TB, Veno MT, Kjems J (2018). Circular RNAs in cancer: opportunities and challenges in the field. Oncogene.

[35] Singh V, Jaiswal PK, Ghosh I, Koul HK, Yu X, De Benedetti A (2019). Targeting the TLK1/NEK1 DDR axis with Thioridazine suppresses outgrowth of androgen independent prostate tumors. Int J Cancer.

[36] De Benedetti A (2012). The tousled-like kinases as guardians of genome integrity. ISRN Mol Biol.

[37] Salmena L, Poliseno L, Tay Y, Kats L, Pandolfi PP (2011). A ceRNA hypothesis: the Rosetta stone of a hidden RNA language?. Cell.

[38] Li J, Zhuang C, Liu Y, Chen M, Chen Y, Chen Z, He A, Lin J, Zhan Y, Liu L, Xu W, Zhao G, Guo Y, Wu H, Cai Z, Huang W (2016). Synthetic tetracycline-controllable shRNA targeting long non-coding RNA HOXD-AS1 inhibits the progression of bladder cancer. J Exp Clin Cancer Res.

[39] Bossi L, Figueroa-Bossi N (2016). Competing endogenous RNAs: a target-centric view of small RNA regulation in bacteria. Nat Rev Microbiol.

[40] Zhong Y, Du Y, Yang X, Mo Y, Fan C, Xiong F, Ren D, Ye X, Li C, Wang Y, Wei F, Guo C, Wu X, Li X, Li Y, Li G, Zeng Z, Xiong W (2018). Circular RNAs function as ceRNAs to regulate and control human cancer progression. Mol Cancer.

[41] Chen X, Chen RX, Wei WS, Li YH, Feng ZH, Tan L, Chen JW, Yuan GJ, Chen SL, Guo SJ, Xiao KH, Liu ZW, Luo JH, Zhou FJ, Xie D (2018). PRMT5 circular RNA promotes metastasis of urothelial carcinoma of the bladder through sponging miR-30c to induce epithelial-mesenchymal transition. Clin Cancer Res.

[42] Han D, Li J, Wang H, Su X, Hou J, Gu Y, Qian C, Lin Y, Liu X, Huang M, Li N, Zhou W, Yu Y, Cao X (2017). Circular RNA circMTO1 acts as the sponge of microRNA-9 to suppress hepatocellular carcinoma progression. Hepatology.

[43] Lu Q, Liu T, Feng H, Yang R, Zhao X, Chen W, Jiang B, Qin H, Guo X, Liu M, Li L, Guo H (2019). Circular RNA circSLC8A1 acts as a sponge of miR-130b/miR-494 in suppressing bladder cancer progression via regulating PTEN. Mol Cancer.

[44] Memczak S, Jens M, Elefsinioti A, Torti F, Krueger J, Rybak A, Maier L, Mackowiak SD, Gregersen LH, Munschauer M, Loewer A, Ziebold U, Landthaler M, Kocks C, le Noble F, Rajewsky N (2013). Circular RNAs are a large class of animal RNAs with regulatory potency. Nature.

[45] Niu J, Li Z, Li F. Overexpressed microRNA-136 works as a cancer suppressor in gallbladder cancer through suppression of JNK signaling pathway via inhibition of MAP2K4. Am J Physiol Gastrointest Liver Physiol. 2019;317:G670–G681.10.1152/ajpgi.00055.201931369289

[46] Jeong JY, Kang H, Kim TH, Kim G, Heo JH, Kwon AY, Kim S, Jung SG, An HJ (2017). MicroRNA-136 inhibits cancer stem cell activity and enhances the anti-tumor effect of paclitaxel against chemoresistant ovarian cancer cells by targeting Notch3. Cancer Lett.

[47] Li B, Zhou J, Liu P, Hu J, Jin H, Shimono Y, Takahashi M, Xu G (2007). Polycomb protein Cbx4 promotes SUMO modification of de novo DNA methyltransferase Dnmt3a. Biochem J.

[48] Ismail IH, Gagne JP, Caron MC, McDonald D, Xu Z, Masson JY, Poirier GG, Hendzel MJ (2012). CBX4-mediated SUMO modification regulates BMI1 recruitment at sites of DNA damage. Nucleic Acids Res.

[49] Jiao HK, Xu Y, Li J, Wang W, Mei Z, Long XD, Chen GQ (2015). Prognostic significance of Cbx4 expression and its beneficial effect for transarterial chemoembolization in hepatocellular carcinoma. Cell Death Dis.

[50] Li J, Xu Y, Long XD, Wang W, Jiao HK, Mei Z, Yin QQ, Ma LN, Zhou AW, Wang LS, Yao M, Xia Q, Chen GQ (2014). Cbx4 governs HIF-1alpha to potentiate angiogenesis of hepatocellular carcinoma by its SUMO E3 ligase activity. Cancer Cell.

[51] Zeng JS, Zhang ZD, Pei L, Bai ZZ, Yang Y, Yang H, Tian QH (2018). CBX4 exhibits oncogenic activities in breast cancer via Notch1 signaling. Int J Biochem Cell Biol.

